The article "Isolated Polycystic Liver Disease: A Rare Genetic Disorder" was retracted in 2024. Reasons: false authorship; unreliable results or conclusions; no approval from an author; concerns about the authorship.

# Isolated Polycystic Liver Disease: A Rare Genetic Disorder

**DOI:** 10.7759/cureus.18560

**Published:** 2021-10-07

**Authors:** Habib Y Aldabbab, Moayad A Hakeem, Fatimah M Alanazi, Mohammed A Asiri, Mohammad F Al Hani, Rahaf I Alshareef, Abeer R Alkahtani, Rahaf F Alfadhli, Lama Y Alharbi, Abdulla A Jan, Mohanned M Alraddadi, Malak Alshammari

**Affiliations:** 1 College of Medicine, King Faisal University, Al-Ahsa, SAU; 2 College of Medicine, University of Jeddah, Jeddah, SAU; 3 College of Medicine, Northern Border University, Arar, SAU; 4 College of Medicine, King Saud University, Riyadh, SAU; 5 Internal Medicine, Ras Tanura General Hospital, Ras Tanura, SAU; 6 College of Medicine, Imam Mohammad Ibn Saud Islamic University, Riyadh, SAU; 7 College of Medicine, Majmaah University, Al Majma'ah, SAU; 8 College of Medicine, Imam Abdulrahman Bin Faisal University, Dammam, SAU

**Keywords:** case report, genetic disorder, hematemesis, abdominal pain, polycystic liver disease

## Abstract

Polycystic liver disease is a rare clinical condition that causes portal hypertension. It constitutes a group of disorders with liver lesions resulting from abnormal development of the embryological ductal system. Isolated polycystic disease with the absence of polycystic kidney disease is considered a rare condition. We present the case of a 46-year-old man who presented with epigastric pain and episodes of hematemesis. Abdominal examination revealed enlarged liver. He underwent a computed tomography scan that revealed innumerable cystic liver lesions with the presence of ascites. Further investigations confirmed abnormal liver functions and portal hypertension. Physicians need to consider this diagnosis in the appropriate clinical settings. Extensive involvement of the liver may lead to persistent severe symptoms requiring liver transplantation.

## Introduction

Epigastric abdominal pain is a common complaint in the emergency department. It typically includes common cardiac, hepatic, biliary, and pancreatic etiologies. However, polycystic liver disease is a rare clinical condition that causes portal hypertension. It constitutes a group of disorders with liver lesions resulting from abnormal development of the embryological ductal system. Polycystic liver disease is usually due to autosomal dominant conditions in adults [1]. However, isolated polycystic disease is rare. Herein, we presented the case of a middle-aged man who presented with epigastric pain and episodes of hematemesis that were eventually diagnosed as isolated polycystic liver disease.

## Case presentation

A 46-year-old man presented to the emergency department with abdominal pain for a one-week duration. He reported that the pain was gradually increasing in intensity. The pain was diffuse but mainly located in the epigastrium. It was constant pain and associated with decreased appetite, abdominal distension, and recurrent episodes of vomiting that contains blood. He did not report a report any change in bowel or urinary habits. His past surgical history included a laparoscopic appendectomy; otherwise, he was healthy and did not experience any health issues. He does not drink alcohol or smoke cigarettes. There was no history of liver diseases in the family.

The article "Isolated Polycystic Liver Disease: A Rare Genetic Disorder" was retracted in 2024. Reasons: false authorship; unreliable results or conclusions; no approval from an author; concerns about the authorship.

On examination, the patient was alert, conscious, and oriented. The general examination appeared normal. His vital signs were as follows: temperature of 37.2℃, heart rate of 120 bpm, respiratory rate of 18 bpm, and blood pressure of 112/70 mmHg. Abdominal examination revealed a distended abdomen with an enlarged liver span. Further, he was noted to have moderate ascites. Cardiorespiratory examination revealed normal findings. Laboratory findings revealed a mild elevation in the liver enzymes with an aspartate transaminase level of 51 U/L and an alanine transaminase level of 67 U/L. The albumin level was 2.9 g/dL and the bilirubin level was 1.3 g/dL. The blood glucose level was within the normal limits. Hematological and other biochemical investigations revealed normal findings (Table 1).

**Table 1:** Summary of the results of laboratory findings

Laboratory Investigation	Unit	Result	Reference Range
Hemoglobin	g/dL	13.1	13.0–18.0
White Blood Cell	1000/mL	8.2	4.0–11.0
Platelet	1000/mL	340	140–450
Erythrocyte Sedimentation Rate	mm/hr.	19	0–20
C-Reactive Protein	mg/dL	8.3	0.3–10.0
Total Bilirubin	mg/dL	1.3	0.2–1.2
Albumin	g/dL	2.9	3.4–5.0
Alkaline Phosphatase	U/L	50	46–116
Gamma-Glutamyltransferase	U/L	45	15–85
Alanine Transferase	U/L	67	14–63
Aspartate Transferase	U/L	51	15–37
Lactate Dehydrogenase	U/L	150	140–280
Blood Urea Nitrogen	mg/dL	17	7–18
Creatinine	mg/dL	1.1	0.7–1.3
Sodium	mEq/L	136	136–145
Potassium	mEq/L	3.6	3.5–5.1
Chloride	mEq/L	105	98–107
D-Dimer	ng/mL	400	220–500
Prothrombin Time	sec	13.0	11–13.5
Partial Thromboplastin Time	sec	30	25–35

The patient underwent abdominal ultrasound examination, which showed an enlarged liver with diffuse multiple cysts. The patient was resuscitated with intravenous fluid hydration. Subsequently, he underwent a computed tomography scan of the abdomen, which revealed innumerable, homogeneous, and hypoattenuating cystic lesions in the liver (Figure 1). The portal vein measures 23 mm in diameter. Both kidneys were normal. Given the extensive cystic disease, the patient was referred to a hepatology center for possible liver transplantation.

**Figure 1:** Computed tomography Computed tomography image showing innumerable, homogeneous, and hypoattenuating cystic lesions in the liver (L) along with ascites (asterisk)

The article "Isolated Polycystic Liver Disease: A Rare Genetic Disorder" was retracted in 2024. Reasons: false authorship; unreliable results or conclusions; no approval from an author; concerns about the authorship.

## Discussion

We presented the case of a middle-aged man with isolated polycystic liver disease presenting with abdominal pain and hematemesis. In this condition, the hepatic involvement ranges from limited areas of cystic disease to diffuse hepatic involvement of all segments of the liver. It is an autosomal dominant condition resulting in malformation of the ductal plate of the small intrahepatic ducts. However, there was no family history of liver disease in the family indicating a sporadic form of polycystic liver disease. It is reported that up to 50% of cases are related to mutations in the PRKCSH or SEC63 genes [2].

Several anomalies have been described in patients with polycystic liver disease. These anomalies include biliary hamartoma, Caroli disease, and polycystic kidney disease [3]. In the present case, however, the patient did not have any other association. The typical presentation of polycystic liver disease includes a non-specific, dull abdominal pain, abdominal dimension, shortness of breath, and early satiety. Such symptoms were present in our case. Additionally, the polycystic liver can exert extrinsic compression of the portal vein resulting in portal hypertension. Polycystic liver disease is more prevalent among women. Further, pregnancy and exogenous estrogen use are considered risk factors for this disorder. Hence, some hypotheses suggest a possible hormonal role in the pathogenesis of liver cysts.

The management options for polycystic liver disease include medical and surgical approaches. The medical approaches include the use of somatostatin analogs to decrease the size of the hepatic cysts [4]. Additionally, percutaneous aspiration of the cysts may be used. Total hepatectomy or liver transplantation may be considered in severe cases [5]. Generally, patients with polycystic liver disease have a good prognosis and do not exhibit the typical liver cirrhosis pathway. The indication of liver transplantation for these patients is generally related to the severity of symptoms and their impact on the quality of life of patients.

The presence of liver cysts along with elevated glucose levels should raise the suspicion of the maturity-onset diabetes of the young (MODY). In type 5, there is a mutation in the HFN1B gene, which plays a key role in the development of multiple organs, including the kidneys, liver, and pancreas. Patients with MODY5 may have pancreatic dysfunction, liver disease, and renal cysts [6].

## Conclusions

Isolated polycystic liver disease is a rare clinical entity. Physicians need to consider this diagnosis in patients with abdominal pain, ascites, and enlarged liver, even in the absence of a family history of liver disease. Extensive involvement of the liver may lead to refractory symptoms requiring liver transplantation.
